The article "Thermal Radiation Effect on Unsteady Magneto-Convective Heat-Mass Transport Passing in a Vertical Permeable Sheet with Chemical Reaction" was published in 2022. Journal: Comput Math Methods Med.

# Thermal Radiation Effect on Unsteady Magneto-Convective Heat-Mass Transport Passing in a Vertical Permeable Sheet with Chemical Reaction

**DOI:** 10.1155/2022/2872940

**Published:** 2022-06-28

**Authors:** Md. Hasanuzzaman, Tanvir Ahamed, Akio Miyara

**Affiliations:** ^1^Department of Mathematics, Khulna University of Engineering & Technology, Khulna 9203, Bangladesh; ^2^Department of Mechanical Engineering, Saga University, Saga-shi 840-8502, Japan; ^3^International Institute for Carbon-Neutral Energy Research, Kyushu University, Fukuoka-shi 819-0395, Japan

## Abstract

The unsteady magneto-convective heat-mass transport passing in a vertical porous sheet with the thermal radiation and the chemical reaction effects has been examined numerically. The governing PDEs have been transferred into ODEs by applying the local similarity transformation. The nondimensional governing equations including the boundary conditions are solved by applying the superposition method with the help of the “MATLAB ODE45” software numerically. The influence of emerging nondimensional numbers/parameters, for example, the Prandtl number (Pr), thermal radiation parameter (*R*), Schmidt number (Sc), and chemical reaction parameter (*K*_r_), on fluid velocity, concentration, and thermal radiation within the boundary layer has been examined. The outcomes indicate that enhancing values of the Soret and Dufour numbers reduce the thermal boundary layer thickness. Uplifting values of the thermal radiation (0.5-3.5) enhance the local skin friction coefficient and mass transfer rate by approximately 15% and 78% but decrease the heat transfer rate by 47%. The local skin friction coefficient enhances about 21%, and the mass transfer rate reduces about 64% due to an increase in the chemical reaction parameter (0.5-2.0). Finally, we compared our numerical results with previously published literature and observed them to have a good agreement.

## 1. Introduction

The MHD (hydromagnetic) free convective and heat transfer flow problems in a permeable medium play an important role in various industrial and scientific processes, for example, problems of boundary layer flow control, plasma studies, thermo nuclear fusion, furnace design, metallurgy, mineral and petroleum engineering, geothermal energy extraction, chemical engineering, and solar power technology. These types of problems act on the different engineering devices applying electrically conducting fluids, for example, MHD generators, plasma jet engines, MHD accelerators, MHD pumps, nuclear reactors, and MHD flow meters. The free magneto-convective heat-mass transport passing a permeable medium restricted by a vertical permeable sheet with constant heat flux has been examined by Raptis and Kafousias [1]. The influences of natural convection and mass transport on the oscillatory flow through a moving vertical isothermal sheet under constant heat sources and suction effects have been explained by Raptis [2]. Sattar [3] discussed the impact of variable suction and Hall current effects on unsteady free magneto-convective heat-mass transport passing a permeable medium near a vertical permeable sheet with constant heat flux. The non-Darcy mixed convective flow along a vertical wall in a saturated permeable medium has been analyzed by Lai and Kulacki [4]. Many researchers such as Eckert and Drake [5], Pop and Ingham [6], Nield and Bejan [7], Gebhart et al. [8], and Incropera et al. [9] had well documented the comprehensive studies of free convective boundary layer flow over different geometrical bodies with heat and mass transfer in nonpermeable media. Hydromagnetic (MHD) manages the heat and force exchanged by the surface in boundary layer flow problems. Srinivas and Muthuraj [10] debilitated the homotopy analysis technique to get an approximate solution for the hydromagnetic viscous incompressible fluid flow under the permeability and thermal radiation effects. The MHD viscoelastic fluid characteristic passing a wall has been investigated by Raftari and Vajravelu [11]. Si et al. [12] explored the heat transfer for micropolar fluid embedded in a porous medium. Convective flows with simultaneous mass and heat transfer with the effect of the chemical reaction and a magnetic field rise in numerous transport processes both artificially and naturally in various engineering and science applications. This concept plays a significant part in the chemical industry, cooling and power drying industry, cooling of nuclear reactors, chemical vapor deposition on surfaces, petroleum industries, etc. Free convective flow happens frequently in nature. It happens owing to concentration distinctions and owing to temperature differences or the combination of these two, such that there exists differences in water mass and in atmospheric flows, and therefore, the flow is affected by such mass distinction. Nield and Bejan [7] explained the flow past and through permeable media in detail. Hiremath and Patil [13] discussed the influence of free or natural convective flows on the oscillatory flow passing in a permeable medium. At constant temperature, the free convection currents are bounded by a vertical plane surface. Sharma et al. [14] explained the fluctuating mass and heat transfer on three-dimensional flow past a permeable medium with the variable permeability effect. Howell et al. [15] explained that when technological methods take space, then the thermal radiation heat transfer has become so significant at higher temperatures. The impact of thermal radiation heat transfer cannot be ignored. MHD flow, mass, and heat transfer become more momentous in industrial areas with thermal radiation effects. Various methods in science and engineering sides happen at high temperatures. The concept of heat transfer of the thermal radiation becomes very notable for the model of the relevant instruments. The final product quality is dependent on the heat-controlling factors to a great extent. The idea of radiative heat transfer in the process may be conducted to the wished-for product with sought qualities. The impact of thermal radiation on unsteady magneto-convective heat-mass transport passing in a permeable space has been analyzed by Olanrewaju [16]. In many practical applications in the presence of two forms of chemical effects such as heterogeneous and homogeneous, the heterogeneous and homogeneous reaction mass transfer takes space by diffusive operations. These reactions include the species' molecular diffusion. A heterogeneous reaction takes space within the phase boundary or in a limited area. But a homogeneous reaction is similar to an internal source of heat generation. It happens uniformly throughout a given phase. The concentration is directly proportional to the rate of reaction in the chemical reaction with the first order. The diffusive species may be generated or absorbed due to various types of chemical reactions in the presence of the ambient fluid. It may be greatly influenced by the quality and properties of completed products. The impact of chemical reaction and magnetic field on unsteady natural convection fluid flow passing in a vertical porous sheet under the diffusion-thermo and thermal-diffusion impacts has been explained by Reddy et al. [17]. Further, Raju [18] has observed the impact of the transverse magnetic field on an unsteady free convection flow past a vertical sheet. He also explained the numerical outcomes for the impacts of thermal-diffusion and diffusion-thermo on their system with heat sources and thermal radiation effects. Sharma and Bhaskar [19] investigated the impacts of thermal radiation and chemical reaction on the three-dimensional MHD incompressible and viscous flow. They also considered the Dufour and Soret impacts on their system. The impact of the magnetic field and thermal radiation on a transient natural convective nanofluid that streams along with a vertical sheet has been analyzed by Kumar et al. [20]. Daniel et al. [21] explained the combined viscous dissipation effects, Joule heating, and thermal radiation on the steady two-dimensional electrical MHD boundary layer nanofluid flow over a porous linear stretching sheet. Also, they have used the Keller box method for solving the coupled ODEs.

With the combination of mass and heat transfer procedures, the flow is run by density differences created by concentration gradient, temperature gradient, and material composition simultaneously. The Dufour (diffusion-thermo) effect is the concentration differences which create the energy flux. The Soret (thermal-diffusion) effect is the temperature gradient which creates the mass flux. The Soret influence, for example, has been used in mixture and for isotope separation between gases with medium molecular weight and gases with very light molecular weight. The Dufour and Soret influences are faced in numerous practical applications, for example, in the fields of chemical engineering and geosciences. The effects of the Dufour number and Soret number on the hydromagnetic mixed convection-radiation interaction along a porous surface submerged in a permeable medium have been studied by Chamkha and Ben-Nakhi [22]. Alam and Rahman [23] discussed the influence of Dufour and Soret effects on steady hydromagnetic free convective heat and mass transfer flow through a vertical permeable sheet embedded in a permeable medium. Alam et al. [24] explained the Soret and Dufour effects on unsteady free convective and mass flow through an impulsively started infinite vertical porous flat sheet in a porous medium. They also used in their simulation the transversely applied magnetic field effect. The impacts of Hall currents, thermal radiation, and Dufour and Soret on MHD flow by mixed convective heat flow over a vertical surface in permeable media have been investigated by Shateyi et al. [25]. They have found the numerical solutions of this problem by using MATLAB routine bvp4c. Hasanuzzaman et al. [26] explained the effect of transpiration on unsteady free convective and heat transfer flow around a vertical slender body. They have also used the shooting technique for solving the ODEs with the help of “MATLAB ODE45” software. Their simulation is almost the same as our simulation. Hasanuzzaman et al. [27] investigated the unsteady free magneto-convective heat-mass transport passing in an infinite vertical permeable sheet in the presence of Dufour and thermal diffusion effects.

The main result of this current research is to suppose the above problems passing a vertical permeable sheet taking into account the chemical reaction and thermal radiation effects. The mail novelty of this study is to compare our results with a published paper. Another novelty of this paper is also enhanced by assuming the chemical reaction and thermal radiation under the Runge-Kutta-Merson integration technique which is not explained yet. Computations have been performed for a vast range of the dimensionless numbers/parameters; for example, thermal radiation parameter, Soret number, suction parameter, chemical reaction parameter, Prandtl number, Dufour number, Schmidt number, and magnetic number on temperature, concentration, and velocity profiles are discussed graphically and analyzed. Besides, the properties of the heat and mass transfer and skin friction coefficient have been explained in the tabular forms.

## 2. Governing Equations

The two-dimensional unsteady free magneto-convective heat-mass transport of an electrically conducting viscous fluid passing in a vertical permeable sheet at *y* = 0 is considered. The direction of an upward sheet is the *x*-axis. The *y*-axis is the normal of the plane sheet in the fluid. When a uniform magnetic field **B** is imposed on the sheet, then the permeable sheet is supposed to be electrically nonconducting along the *y*-axis as shown in Figure 1.

We presume that the induced magnetic field is insignificant for a very small flow magnetic Reynolds number compared with one of the research projects [28]. Then, the lines of the magnetic force are permanent relative to the fluid such that **B** = (0, *B*_0_, 0). The current density is **J** = (*J*_*x*_, *J*_*y*_, *J*_*z*_), and the continuity equation of charge is ∇.**J** = 0 which implies that *J*_*y*_ = constant. The propagation direction is presumed only along the *y*-axis. This propagation direction does not have any change along the *y*-axis. So the differentiation of *J*_*y*_ with respect to *y* must be zero such as *∂J*_*y*_/*∂y* = 0. Since this constant of integration is zero when the sheet is electrically nonconducting, *J*_*y*_ = 0 at the sheet and it is zero everywhere.

The one-dimensional problem under the Boussinesq approximation and the above assumptions may be used in the below form [24]:

The continuity equation:

(1) $$\begin{array}{c} \frac{\partial v}{\partial y}=0. \end{array}$$

The momentum equation:

(2) $$\begin{array}{c} \frac{\partial u}{\partial t}+v\frac{\partial u}{\partial y}=\upsilon \frac{\partial^{2}u}{\partial y^{2}}+g\beta \left(T-T_{\infty }\right)+g\beta^{*}\left(C-C_{\infty }\right)-\frac{\sigma^{\prime }B_{0}^{2}u}{\rho }. \end{array}$$

The energy equation:

(3) $$\begin{array}{c} \frac{\partial T}{\partial t}+v\frac{\partial T}{\partial y}=\frac{k}{\rho C_{p}}\frac{\partial^{2}T}{\partial y^{2}}+\frac{D_{\text{m}}k_{T}}{C_{\text{s}}C_{p}}\frac{\partial^{2}C}{\partial y^{2}}-\frac{1}{\rho C_{p}}\frac{\partial q_{r}}{\partial y}. \end{array}$$

The concentration equation:

(4) $$\begin{array}{c} \frac{\partial C}{\partial t}+v\frac{\partial C}{\partial y}=D_{\text{m}}\frac{\partial^{2}C}{\partial y^{2}}+\frac{D_{\text{m}}k_{T}}{T_{\text{m}}}\frac{\partial^{2}T}{\partial y^{2}}+K^{\prime }\left(C-C_{\infty }\right). \end{array}$$

The boundary conditions are given by

(5) $$\begin{array}{c} t>0,u=U_{0}\left(t\right),v=v\left(t\right),T=T_{\text{w}},C=C_{\text{w}}\text{ at }y=0, \end{array}$$

(6) $$\begin{array}{c} t>0,u=0,v=0,T⟶T_{\infty },C⟶C_{\infty }\text{ at }y⟶\infty , \end{array}$$

where *u* and *v* are the components of the velocity in the *x* and *y* directions, respectively. The fluid density is *ρ*, *υ* is the kinematic viscosity, the coefficient of concentration expansion is *β*^∗^, the coefficient of thermal expansion is *β*, the fluid temperature is *T*, the wall temperature is T_w_, the fluid temperature in the free stream is *T*_∞_, the component of radiative heat flux is *q*_r_, *C* is the fluid concentration, the wall concentration is *C*_w_, the free stream concentration is *C*_∞_, the thermal conductivity of the sheet is *k*, the concentration susceptibility is *C*_s_, the specific heat at constant pressure is *C*_*p*_, the mean temperature of the fluid is *T*_m_, *k*_*T*_ is the thermal diffusion ratio, the mass diffusivity coefficient is *D*_m_, *g* is the gravitational acceleration, and the chemical reaction rate of species concentration is *K*′.

Upon using a similarity parameter *σ*,

(7) $$\begin{array}{c} \sigma =\sigma \left(t\right), \end{array}$$

where the time-dependent length scale is *σ*. The solution of equation (1) is supposed in terms of this length scale given by

(8) $$\begin{array}{c} v=-v_{0}\frac{\upsilon }{\sigma }. \end{array}$$

Here, the dimensionless normal velocity at the sheet is *v*_0_. *v*_0_ < 0 represents blowing, and *v*_0_ > 0 represents suction.

According to the Rosseland approximation [29], the radiative heat flux *q*_r_ is given by

(9) $$\begin{array}{c} q_{\text{r}}=-\frac{4\sigma^{*}}{3K^{*}}\frac{\partial T^{4}}{\partial y}, \end{array}$$

where the constant of Stefan-Boltzmann is *σ*^∗^ and the coefficient of the mean absorption is *K*^∗^.

We consider from Raptis [30] that the difference between the fluid temperature and the free stream temperature is small enough.

Expanding in a Taylor series *T*^4^ about *T*_0_ and ignoring higher-order terms, we have

(10) $$\begin{array}{c} T^{4}≅4T_{0}^{3}T-3T_{0}^{4}. \end{array}$$

Now, the below similarity variables can be applied:

(11) $$\begin{array}{c} \eta =\frac{y}{\sigma },f\left(\eta \right)=\frac{u}{U_{0}},\theta \left(\eta \right)=\frac{T-T_{\infty }}{T_{\text{w}}-T_{\infty }},\phi \left(\eta \right)=\frac{C-C_{\infty }}{C_{\text{w}}-C_{\infty }}. \end{array}$$

Applying equations (7)–(11), equations (1)–(4) are converted into the nondimensional coupled ODEs as follows:

(12) $$\begin{array}{c} f^{\prime \prime }+2\xi f^{\prime }+G_{\text{r}}\theta +G_{\text{m}}\phi -Mf=0, \end{array}$$

(13) $$\begin{array}{c} \theta^{\prime \prime }+\frac{\text{Pr}}{1+R}\left(2\xi \theta^{\prime }+\text{Df}\phi^{\prime \prime }\right)=0, \end{array}$$

(14) $$\begin{array}{c} \phi^{\prime \prime }+2\xi \text{Sc}\phi^{\prime }+\text{ScSo}\theta^{\prime \prime }+K_{\text{r}}\phi =0. \end{array}$$

The converted boundary conditions are given by

(15) $$\begin{array}{c} f=1,\theta =1,\phi =1\text{ at }\eta =0, \end{array}$$

(16) $$\begin{array}{c} f=0,\theta =0,\phi =0\text{ at }\eta ⟶\infty , \end{array}$$

where the local Grashof number is *G*_*r*_ = *gβ*(*T*_w_ − *T*_∞_)*σ*^2^/*U*_0_*υ*, the magnetic force parameter is *M* = *σ*′*B*_0_^2^*σ*^2^/*ρυ*, the Prandtl number is Pr = *ρυC*_*p*_/*k*, *G*_m_ = *gβ*^∗^(*C*_w_ − *C*_∞_)*σ*^2^/*U*_0_*υ* is the modified local Grashof number, the Dufour number is *D*_f_ = *D*_m_*k*_*T*_(*C*_w_ − *C*_∞_)/*C*_s_*C*_*p*_*υ*(*T*_w_ − *T*_∞_), the Soret number is *S*_0_ = *D*_m_*k*_*T*_(*T*_w_ − *T*_∞_)/*υT*_m_(*C*_w_ − *C*_∞_), the Schmidt number is Sc = *υ*/*D*_m_, the thermal radiation parameter is *R* = 16*σ*^∗^*T*_W_^2^/3*K*^∗^*K*, the chemical reaction parameter is *K*_r_ = *K*′*σ*^2^/*υ*, and *ξ* = *η* + (*v*_0_/2).

The flow parameters are the skin-friction coefficient (*τ*), the Nusselt number (*Nu*), and the local Sherwood number (Sh) which are defined as

(17) $$\begin{array}{c} \tau \propto f^{\prime },\text{Nu}\propto -\theta^{\prime },\text{Sh}\propto -\phi^{\prime }. \end{array}$$

## 3. Numerical Solution

By applying the superposition method [31], the solutions of equations (12)–(14) with the boundary conditions (15)–(16) are obtained. The boundary value problems are converted into the initial value problem by using the superposition technique. This initial value problem may easily be integrated by using an initial value solver. So to convert equations (12)–(14) to an initial value problem, the functions *f*(*η*), *θ*(*η*), and *ϕ*(*η*) are, respectively, decomposed to

(18) $$\begin{array}{c} f\left(\eta \right)=f_{1}\left(\eta \right)+\mu f_{2}\left(\eta \right)+\lambda f_{3}\left(\eta \right)+\delta f_{4}\left(\eta \right), \end{array}$$

(19) $$\begin{array}{c} \theta \left(\eta \right)=\theta_{1}\left(\eta \right)+\mu \theta_{2}\left(\eta \right)+\lambda \theta_{3}\left(\eta \right)+\delta \theta_{4}\left(\eta \right), \end{array}$$

(20) $$\begin{array}{c} \phi \left(\eta \right)=\phi_{1}\left(\eta \right)+\mu \phi_{2}\left(\eta \right)+\lambda \phi_{3}\left(\eta \right)+\delta \phi_{4}\left(\eta \right), \end{array}$$

where *δ*, *μ*, and *λ* are arbitrary constants. Now, putt equations (18)–(20) in equations (12)–(14) and then separate the various coefficients to zero. Finally, we get the differential equations which are given by

(21) $$\begin{array}{c} f_{1}^{\prime \prime }+2\xi f_{1}^{\prime }-Mf_{1}+G_{r}\theta_{1}+G_{\text{m}}\phi_{1}=0,\\ f_{2}^{\prime \prime }+2\xi f_{2}^{\prime }-Mf_{2}+G_{r}\theta_{2}+G_{\text{m}}\phi_{2}=0,\\ f_{3}^{\prime \prime }+2\xi f_{3}^{\prime }-Mf_{3}+G_{r}\theta_{3}+G_{\text{m}}\phi_{3}=0,\\ f_{4}^{\prime \prime }+2\xi f_{4}^{\prime }-Mf_{4}+G_{r}\theta_{4}+G_{\text{m}}\phi_{4}=0,\\ \theta_{1}^{\prime \prime }+\frac{\text{Pr}}{1+R}\left(2\xi \theta_{1}^{\prime }+\text{Df}\phi_{1}^{\prime \prime }\right)=0,\\ \theta_{2}^{\prime \prime }+\frac{\text{Pr}}{1+R}\left(2\xi \theta_{2}^{\prime }+\text{Df}\phi_{2}^{\prime \prime }\right)=0,\\ \theta_{3}^{\prime \prime }+\frac{\text{Pr}}{1+R}\left(2\xi \theta_{3}^{\prime }+\text{Df}\phi_{3}^{\prime \prime }\right)=0,\\ \theta_{4}^{\prime \prime }+\frac{\text{Pr}}{1+R}\left(2\xi \theta_{4}^{\prime }+\text{Df}\phi_{4}^{\prime \prime }\right)=0,\\ \phi_{1}^{\prime \prime }+2\xi \text{Sc}\phi_{1}^{\prime }+\text{ScSo}\theta_{1}^{\prime \prime }+K_{\text{r}}\phi_{1}=0,\\ \phi_{2}^{\prime \prime }+2\xi \text{Sc}\phi_{2}^{\prime }+\text{ScSo}\theta_{2}^{\prime \prime }+K_{\text{r}}\phi_{2}=0,\\ \phi_{3}^{\prime \prime }+2\xi \text{Sc}\phi_{3}^{\prime }+\text{ScSo}\theta_{3}^{\prime \prime }+K_{\text{r}}\phi_{3}=0,\\ \phi_{4}^{\prime \prime }+2\xi \text{Sc}\phi_{4}^{\prime }+\text{ScSo}\theta_{4}^{\prime \prime }+K_{\text{r}}\phi_{4}=0. \end{array}$$

The initial values of the decomposed functions *f*_1_(*η*), *f*_2_(*η*), *f*_3_(*η*), *f*_4_(*η*), ⋯ are now got passing in the boundary conditions (15) and (16) as

(22) $$\begin{array}{c} f_{1}\left(\eta \right)=1.0,f_{2}\left(\eta \right)=0,f_{3}\left(\eta \right)=0,f_{4}\left(\eta \right)=0,\\ \theta_{1}\left(\eta \right)=1.0,\theta_{2}\left(\eta \right)=0,\theta_{3}\left(\eta \right)=0,\theta_{4}\left(\eta \right)=0,\\ \phi_{1}\left(\eta \right)=1.0,\phi_{2}\left(\eta \right)=0,\phi_{3}\left(\eta \right)=0,\phi_{4}\left(\eta \right)=0. \end{array}$$

Also, as  *η*⟶∞, using the boundary conditions (15) and (16) in (16)–(18), we obtain

(23) $$\begin{array}{c} \mu =-\frac{f_{1}\left(\theta_{3}\phi_{4}-\theta_{4}\phi_{3}\right)+\theta_{1}\left(f_{4}\phi_{3}-f_{3}\phi_{4}\right)+\phi_{1}\left(f_{1}\theta_{4}-f_{4}\theta_{1}\right)}{f_{2}\left(\theta_{3}\phi_{4}-\theta_{4}\phi_{3}\right)+f_{1}\left(f_{4}\phi_{3}-f_{3}\phi_{4}\right)+\phi_{1}\left(f_{1}\theta_{4}-f_{4}\theta_{1}\right)},\\ \lambda =-\frac{f_{1}\left(\theta_{4}\phi_{2}-\theta_{2}\phi_{4}\right)+\theta_{1}\left(f_{2}\phi_{4}-f_{4}\phi_{2}\right)+\phi_{1}\left(\theta_{2}f_{4}-\theta_{4}f_{2}\right)}{f_{2}\left(\theta_{3}\phi_{4}-\theta_{4}\phi_{3}\right)+f_{1}\left(f_{4}\phi_{3}-f_{3}\phi_{4}\right)+\phi_{1}\left(f_{1}\theta_{4}-f_{4}\theta_{1}\right)},\\ \delta =-\frac{f_{1}\left(\theta_{2}\phi_{3}-\theta_{3}\phi_{2}\right)+\theta_{1}\left(f_{3}\phi_{2}-f_{2}\phi_{3}\right)+\phi_{1}\left(\theta_{3}f_{2}-\theta_{2}f_{3}\right)}{f_{2}\left(\theta_{3}\phi_{4}-\theta_{4}\phi_{3}\right)+f_{1}\left(f_{4}\phi_{3}-f_{3}\phi_{4}\right)+\phi_{1}\left(f_{1}\theta_{4}-f_{4}\theta_{1}\right)}. \end{array}$$

In (16)–(18), all the functional values are obtained as

(24) $$\begin{array}{c} \frac{\partial f\left(\eta \right)}{\partial \eta }=\frac{\partial f_{1}\left(\eta \right)}{\partial \eta }+\mu \frac{\partial f_{2}\left(\eta \right)}{\partial \eta }+\lambda \frac{\partial f_{3}\left(\eta \right)}{\partial \eta }+\delta \frac{\partial f_{4}\left(\eta \right)}{\partial \eta },\\ \frac{\partial \theta \left(\eta \right)}{\partial \eta }=\frac{\partial \theta_{1}\left(\eta \right)}{\partial \eta }+\mu \frac{\partial \theta_{2}\left(\eta \right)}{\partial \eta }+\lambda \frac{\partial \theta_{3}\left(\eta \right)}{\partial \eta }+\delta \frac{\partial \theta_{4}\left(\eta \right)}{\partial \eta },\\ \frac{\partial \phi \left(\eta \right)}{\partial \eta }=\frac{\partial \phi_{1}\left(\eta \right)}{\partial \eta }+\mu \frac{\partial \phi_{2}\left(\eta \right)}{\partial \eta }+\lambda \frac{\partial \phi_{3}\left(\eta \right)}{\partial \eta }+\delta \frac{\partial \phi_{4}\left(\eta \right)}{\partial \eta }. \end{array}$$

The missing slopes are given by

(25) $$\begin{array}{c} \frac{\partial f\left(0\right)}{\partial \eta },\frac{\partial \theta \left(0\right)}{\partial \eta },\frac{\partial \phi \left(0\right)}{\partial \eta }. \end{array}$$

Now, assuming the values of the missing slopes:

(26) $$\begin{array}{c} \frac{\partial f\left(0\right)}{\partial \eta }=\mu ,\frac{\partial \theta \left(0\right)}{\partial \eta }=\lambda ,\frac{\partial \phi \left(0\right)}{\partial \eta }=\delta , \end{array}$$

the initial conditions for the missing slopes of the decomposed functions are observed easily. Integrate equations (12)–(14) by using an initial value solver to get the converged solutions which are focused graphically in Figures 2–15 by applying the Runge-Kutta-Merson integration scheme. Now, Sh, Nu, and *τ* are, respectively, denoted as the Sherwood number, the Nusselt number, and the local skin friction coefficient which are proportionate to −*∂ϕ*(0)/*∂η*, −*∂θ*(0)/*∂η*, and *∂f*(0)/*∂η*, respectively.

## 4. Results and Discussions

The impact of thermal radiation on unsteady magneto-convective heat-mass transport passing in a vertical permeable sheet under the chemical reaction effect has been analyzed numerically in this research. By applying the superposition technique, we have solved the set ODEs (10)–(12) with the boundary conditions (15) and (16) numerically. Also, we have used the “MATLAB ODE45” software. The impacts of the suction parameter (*v*_0_), the Dufour number (Df), the magnetic force parameter (*M*), the Soret number (So), the radiation parameter (*R*), the Schmidt number (Sc), the chemical reaction parameter (*K*_r_), and the Prandtl number (Pr) on temperature, concentration, and velocity distributions are displayed in Figures 2–15. The values 7.0, 1.0, and 0.71 are supposed for Pr (1.0 and 7.0 for water at 17^0^ and 0.71 for air at 20^0^). The values 0.75, 0.60, and 0.22 are also supposed for Sc (0.60 for vapor water, 0.22 for hydrogen, and 0.75 for oxygen). The remaining nondimensional parameter/number values are however taken arbitrarily.

### 4.1. Velocity Distributions for Various Values of Numbers/Parameters

Figure 2 depicts the velocity distribution for various values of the magnetic force parameter (*M*). From Figure 2, it is found that the fluid velocity reduces for rising values of magnetic parameter (*M*). With increasing values of the magnetic force parameter, a resistive kind of force, for example, a drag force, is generated. This resistive type of force is called Lorentz force. This is due to the fact that the magnetic force parameter produces a resistive kind of force (Lorentz force) which causes reduction in the fluid velocity.  Figure 3 represents the impact of the suction parameter (*v*_0_) on the velocity profile. When *v*_0_ > 0, then the whole system fluid suction event has happened. It can be concluded from Figure 3 that for the case of suction (*v*_0_ > 0), the mass of the fluid in the computational domain decreases. For this reason, the frictional force reduces. So the velocity of fluid reduces for increasing values of the suction. This is because suction stabilizes the boundary layer growth. The velocity distribution is observed to enhance and reaches the highest value in a region close to the leading edge of the sheet and then reduces to zero gradually. The Prandtl number (Pr = *ρυC*_*p*_/*k*) is the proportional to the kinematic viscosity. From graph 4, it is noticed that when the Prandtl number enhances, then the fluid kinematic viscosity increases. For this reason, the fluid particles cannot move freely. So the fluid velocity reduces. Physically, due to enhancement of the Prandtl number (Pr), the kinematic viscosity of the fluid increases which in turn makes the fluid much thicker. For this reason, the velocity of the fluid reduces. The behavior of thermal radiation parameter (*R*) on the velocity distribution is displayed in Figure 5. The thermal radiation parameter is defined as *R* = (16*σ*^∗^*T*_W_^2^)/(3*k*^∗^*k*) and shaped in the increased thermal diffusion term in equation (13), i.e., 1/Pr(1 + *R*)*θ*^″^(*η*). The comparative contribution of the thermal radiation heat transfer to the thermal conduction heat transfer is defined by the thermal radiation parameter. The thermal radiation dominates over thermal conduction when *R* > 1, but the thermal conduction dominates for *R* < 1. The thermal radiation contributions and thermal conduction both are equal for *R* = 1.

We constrict attention to the case of *R* > 1 for the present simulations. Figure 5 expresses that there is a strong acceleration in the linear velocity with enhancing *R*. The energizing of the flow increases thermal diffusion and then decreases momentum diffusion. This leads to a decrease in the thickness of the momentum boundary layer.  Figure 6 illustrates the response of the velocity profile to various values of the Schmidt number (Sc). The Schmidt number is proportional to the kinematic viscosity (*υ*). From graph 6, it is found that when the Schmidt number enhances, then the kinematic viscosity of the fluid increases. For this reason, the fluid particles cannot move freely. So the fluid velocity diminishes. The thickness of the momentum boundary layer is also decreased with a greater Schmidt number.  Figure 8 represents the velocity distribution for various values of the chemical reaction parameter (*K*_r_). The impact of chemical reaction parameter is very momentous in the concentration distribution. Chemical reaction decreases the interfacial mass transfer rate. Reaction enhances the local concentration, hence decreasing its flux and its concentration gradient.

### 4.2. Temperature Distributions for Different Values of Numbers/Parameters

The impact of the suction parameter (*v*_0_) on the temperature distribution is plotted in Figure 8. It is found that with the increasing values of the suction parameter, the fluid temperature reduces. This is due to the fact that the suction parameter decelerates fluid particles through the permeable wall decreasing the growth of the fluid thermal boundary layers. The Prandtl number (Pr) is inversely proportional to the thermal conductivity. The temperature distribution in Figure 9 is found to reduce temperature for uplifting values of Pr (the thermal conductivity decreases). Physically, the lower thermal conductivity has relatively a higher Prandtl number. It reduces heat conduction and so temperature decreases. Hence, the rate of heat transfer enhances for uplifting values of Pr so that the temperature profile lessens.  Figure 10 shows the impact of thermal radiation parameter (*R*) on the temperature profile. From Figure 10, it is noticed that the temperature gradient at the surface decreases for rising values of the thermal radiation parameter. At the surface, the heat transfer rate decreases for increasing *R*. The thermal radiation parameter is accountable for the thermal boundary thickening. The fluid loses the heat energy from the flow region, and for this reason, the system cools. This is due to the fact that the Rosseland approximation increases the temperature.  Figure 11 depicts the effect of diffuso-thermal parameter, i.e., the Dufour number, Df = *D*_m_*k*_*T*_(*C*_w_ − *C*_∞_)/*C*_s_*C*_*p*_*υ*(*T*_w_ − *T*_∞_), on the temperature profile. The Dufour effect mentions heat flux produced by a solutal (concentration) gradient. The temperature distribution accentuates for increasing the diffusion-thermo parameter (Df) as shown in Figure 11. The temperature distribution in the absence of the Dufour effect is smaller in comparison to that in the presence of the Dufour number effect. The thickness of the thermal boundary layer accelerates considerably in the presence of strong Dufour effects.

### 4.3. Concentration Distribution for Various Values of Numbers/Parameters

Figure 12 depicts the impact of the suction parameter (*v*_0_) on the concentration distribution. Sucking decelerated fluid particles past the permeable wall decreases the concentration boundary layer growth.  Figure 13 represents the effect of the various values of the Schmidt number (Sc) on the concentration distribution. The molecular (species) diffusivity is inversely proportional to the Schmidt number. When Sc > 1, then the rate of momentum diffusion exceeds the rate of species diffusion. But it was the opposite behavior for Sc < 1. The concentration (species) and momentum layers will have the same diffusivity rates and thickness for Sc = 1. The concentration distribution in Figure 13 is found to reduce the concentration for uplifting values of Sc. The associated depletion in mass diffusivity outcomes in a small forceful mass transfer decreases concentration levels and also reduces the thickness of the concentration boundary layer. This is because mass transfer uses interplay with the species profile and the velocity field in materials which can be manipulated via the Schmidt number.

Figure 14 represents the influence of the Soret number (thermo-diffusive parameter) on the concentration distribution. The Soret number is defined by So = *D*_m_*k*_*T*_(*T*_w_ − *T*_∞_)/*υT*_m_(*C*_w_ − *C*_∞_); i.e., the Soret number is inversely proportional to the mass diffusivity coefficient (*D*_m_). The Soret effect rises where large heavy molecules and small light molecules separate under a temperature gradient. The Soret number enhancement means that the mass diffusivity coefficient increases. For this reason, the concentration distribution increases significantly as the Soret number increases. This outcome is an important enhancement in concentration boundary layer thickness. The impact of the chemical reaction parameter (*K*_r_) on the concentration profile is displayed in Figure 15. Rising values of the chemical reaction parameter increase the concentration of the fluid.

### 4.4. Heat and Mass Transfer Rates and Local Skin Friction

The authors have investigated not only the velocity, temperature, and concentration fields but also the values of the local skin friction coefficient and heat and mass transfer rates. The authors gave the local skin friction coefficient and mass and heat transfer rates in Tables 1–7.

Tables 1–7 represent the impact of different values of the mentioned parameters/numbers on the values of heat and mass transfer rates and local skin friction coefficient. From Tables 1–7, it is found that the skin friction reduces for uplifting values of the magnetic force parameter, suction parameter, Prandtl number, and Schmidt number but enhances for enhancing values of the thermal radiation parameter, Soret number, and chemical reaction parameter. The heat transfer rate enhances for uplifting values of the suction parameter and Prandtl number, but a reverse trend is found for the thermal radiation parameter. Also, the mass transfer rate enhances for rising values of the suction parameter and thermal radiation parameter but decreases for the Prandtl number, Soret number, Schmidt number, and chemical reaction parameter.

### 4.5. Comparison

The present research results have been compared with Alam et al. [24]. The comparison of the local Sherwood number and the local Nusselt number has been shown in Tables 8 and 9, respectively. From these tables, it is found that the comparisons of the present numerical outcomes show a good agreement with previously published outcomes under the special cases. These comparisons ensure the accuracy and validity of the present research work.

## 5. Conclusions

The unsteady free magneto-convective heat-mass transport passing in a vertical permeable sheet has been analyzed numerically under the thermal radiation and the chemical reaction effects. From the above numerical simulations, the below conclusions can be illustrated:

- The local skin friction enhances about 15%, 13%, 28%, 56%, and 21% due to increasing thermal radiation parameter (0.5-3.5), Soret number (1.0-3.0), local Grashof number (5.0-10.0), modified Grashof number (5.0-10.0), and the chemical reaction parameter (0.5-1.0), respectively. Besides, rising values of the magnetic force number (0.5-4.0), suction parameter (0.5-1.5), Prandtl number (0.71-1.0), and Schmidt number (0.22-1.0) reduce the local skin friction by 48%, 7%, 20%, and 15%, respectively
- Uplifting values of the suction parameter (0.5-1.5) and Prandtl number (0.71-1.0) enhance the heat transfer rate by 64% and 23%, respectively, but decrease about 47% for enhancing the thermal radiation parameter (0.5-3.5)
- The mass transfer rate enhances about 5% due to enhancing the suction parameter (0.0-1.5). Besides, increasing the Soret number (1.0-3.0), Schmidt number (0.22-1.0), and chemical reaction parameter (0.5-2.0) decreases the mass transfer rate by 82%, 14%, and 64%, respectively

The result of this paper can be helpful for suspensions, production of paper, plasma studies, thermo nuclear fusion, furnace design, metallurgy, mineral and petroleum engineering, geothermal energy extraction, chemical engineering, solar power technology, etc.

## Figures and Tables

**Figure 1:** Physical model and coordinate system.

**Figure 2:** Velocity distribution for *M*.

**Figure 3:** Velocity distribution for *v*_*o*._

**Figure 4:** Velocity distribution for Pr.

**Figure 5:** Velocity distribution for *R*.

**Figure 6:** Velocity distribution for Sc.

**Figure 7:** Velocity distribution for *K*_r_.

**Figure 8:** Temperature distribution for *v*_0_.

**Figure 9:** Temperature distribution for Pr.

**Figure 10:** Temperature distribution for *R*.

**Figure 11:** Temperature distribution for Df.

**Figure 12:** Concentration distribution for *v*_*o*_.

**Figure 13:** Concentration distribution for Sc.

**Figure 14:** Concentration distribution for So.

**Figure 15:** Concentration distribution for *K*_r_.

**Table 1:** Local skin friction coefficient and heat and mass transfer rates for various values of the magnetic force parameter (*M*).

*M*	*f*′(0)	−*θ*′(0)	−*φ*′(0)
0.5	10.5661100056450	0.932990523828265	0.212030548746318
1.5	8.57903198196934	0.932990523828265	0.212030548746318
3.0	6.54125888977310	0.932990523828265	0.212030548746318
4.0	5.54642746963431	0.932990523828265	0.212030548746318

**Table 2:** Local skin friction coefficient and heat and mass transfer rates for different values of the suction parameter (*v*_0_).

*v*_0_	*f*′(0)	−*θ*′(0)	−*φ*′(0)
0.0	10.6263717252703	0.776316119591959	0.206942024273498
0.5	10.5661100056450	0.932990523828265	0.212030548746318
1.5	9.87472905951721	1.277715565841730	0.216705313239142
2.5	8.65650988800907	1.654923593722190	0.217101577594609
3.5	7.15171444437728	2.055580811460300	0.219821244380065

**Table 3:** Local skin friction coefficient and heat and mass transfer rates for different values of the Prandtl number (Pr).

Pr	*f*′(0)	−*θ*′(0)	−*φ*′(0)
0.71	10.5661100056450	0.932990523828265	0.212030548746318
1.0	10.1474550375773	1.14348338490675	0.126571701930447
7.0	8.46412529013253	4.09185943257223	-1.13908665092652

**Table 4:** Local skin friction coefficient and heat and mass transfer rates for different values of the radiation parameter (*R*).

*R*	*f*′(0)	−*θ*′(0)	−*φ*′(0)
0.5	10.5661100056450	0.932990523828265	0.212030548746318
1.5	11.2599969462999	0.694552002634953	0.305717248240946
2.5	11.7605822700024	0.574503600647324	0.350935901031615
3.5	12.1549714597407	0.499632592878373	0.378197640492878

**Table 5:** Local skin friction coefficient and heat and mass transfer rates for different values of the Soret number (So).

So	*f*′(0)	−*θ*′(0)	−*φ*′(0)
1.0	9.93577413603443	0.932990523828265	0.359608012618135
2.0	10.5661100056450	0.932990523828265	0.212030548746318
3.0	11.1964458957904	0.932990523828265	0.0644530831837319

**Table 6:** Local skin friction coefficient and heat and mass transfer rates for different values of the Schmidt number (Sc).

Sc	*f*′(0)	−*θ*′(0)	−*φ*′(0)
0.22	10.5661100056450	0.932990523828265	0.212030548746318
0.50	9.61314175800702	0.932990523828265	0.221523388418678
1.00	9.03448079369253	0.932990523828265	0.181886779242937

**Table 7:** Local skin friction coefficient and heat and mass transfer rates for different values of the chemical reaction (*K*_r_).

*K*_r_	*f*′(0)	−*θ*′(0)	−*φ*′(0)
0.5	10.5661100056450	0.932990523828265	0.212030548746318
1.0	11.1164907044352	0.932990523828265	0.075836454608230
1.5	11.8324799143874	0.932990523828265	-0.089346500221726
2.0	12.8169889130888	0.932990523828265	-0.300468126650875

**Table 8:** Comparison of the local Sherwood number (Sh) for different values of So and Df when *R* = 0 and *K*_r_ = 0 [24].

So	Df	Alam et al. [24]	Present results	Persistence of error
		Sh	Sh	Sh
1.0	0.06	0.315615	0.31607639	0.046139
0.5	0.12	0.468128	0.46965549	0.152749
0.4	0.15	0.496002	0.49747809	0.147609
0.2	0.30	0.549515	0.54972859	0.021359
0.1	0.60	0.575236	0.57553013	0.029413

**Table 9:** Comparison of the local Nusselt number(Nu) for different values of So and Df when *R* = 0 and *K*_r_ = 0 [24].

So	Df	Alam et al. [24]	Present results	Persistence of error
		Nu	Nu	Nu
1.0	0.06	1.652241	1.65241042	0.016942
0.5	0.12	1.541984	1.54403130	0.204730
0.4	0.15	1.517881	1.51849539	0.061439
0.2	0.30	1.450355	1.45560581	0.525081
0.1	0.60	1.364561	1.36587384	0.131284

## Data Availability

The datasets generated and/or analyzed during the current study are not publicly available due to the fact that we will use these data when extending our further research but are available from the corresponding author on reasonable request.

## Nomenclature

*u*: Velocity component along the *x*-axis
MHD: Hydromagnetic
*J*: Density of current
*T*_w_: Wall temperature
*C*: Fluid concentration
*C*_∞_: Free stream concentration
*U*_0_(*t*): Uniform surface velocity
*g*: Acceleration due to gravity
*β*: Volumetric expansion coefficient with temperature
*k*: Thermal conductivity
*C*_*p*_: Specific heat at constant pressure
*k*_*T*_: Thermal diffusion ratio
*σ*: Similarity parameter
*G*_*r*_: Local Grashof number
*M*: Magnetic parameter
Df: Dafour number
Sc: Schmidt number
*τ*: Local skin friction coefficient
Sh: Sherwood number
*θ*: Dimensionless temperature
*q*_r_: Radiative heat flux
*R*: Thermal radiation parameter
*v*: Velocity component along the *y*-axis
*B*: Uniform magnetic field
*T*: Temperature of fluid
*T*_∞_: Free stream temperature
*C*_w_: Wall concentration
*ρ*: Fluid density
*v*(*t*): Suction velocity
*υ*: Kinematic viscosity
*β* ^∗^: Volumetric expansion coefficient with concentration
*C*_s_: Concentration susceptibility
*T*_m_: Fluid mean temperature
*D*_m_: Mass diffusivity coefficient
*v*_0_: Suction and blowing
*G*_m_: Modified local Grashof number
Pr: Prandtl number
So: Soret number
*t*: Time
Nu: Nusselt number
*f*′: Dimensionless velocity
*ϕ*: Dimensionless concentration
*K*′: Chemical reaction rate of concentration
*K*_r_: Chemical reaction parameter.
